The article "Analysis of Risk Factors for Pneumonia Death in ICU Environment Based on Logistic Regression" was retracted in 2023. Reasons: signs of a paper mill; suspected computer-generated content; unreliable results or conclusions; lack of ethics approval or compliance.

# Analysis of Risk Factors for Pneumonia Death in ICU Environment Based on Logistic Regression

**DOI:** 10.1155/2022/4865776

**Published:** 2022-09-28

**Authors:** Yongping Ma, Fang He, Fei Ouyang

**Affiliations:** ^1^Wuhan Fourth Hospital, Wuhan, Hubei, China; ^2^Wuhan Fifth Hospital, Wuhan, Hubei, China

## Abstract

**Objective:**

To explore the risk and protect factors for death of pneumonia patients in intensive care unit (ICU), we conducted this logistic regression research.

**Methods:**

We collected demographic and nursing care data for 80 patients form Wuhan fourth hospital, in which 40 patients were dead and the other 40 patients were alive. Difference analysis, Pearson's correlation matrix, and logistic regression were conducted to explore the risk and protective factors for living status of pneumonia patients in ICU.

**Results:**

A total of 40 individuals were dead from pneumonia in ICU. The demographic and nursing information had no difference between death and living groups except age. After that, correlation analysis showed that there were correlations between living status, age, and marriage. Logistic regression showed that age (odds ratio (OR) = 0.94, *P* < 0.05) and no education (OR = 0.21, *P* < 0.05) may be harmful for pneumonia patients living status while high-quality nursing (OR = 2.72, *P* < 0.05) may be helpful for pneumonia patients living status.

**Conclusion:**

High-quality care plays an important role in protecting the survival of patients with pneumonia, and old age and uneducated may be the risk factors for the death of patients with pneumonia.

## 1. Introduction

Pneumonia is an infectious disease. Because of the inflammatory reaction of alveoli, lung stroma, and terminal airway, it can be caused by microbial infection and immune injury [1^,^^2^]. Clinically, there will be dyspnea, shortness of breath, accompanied by dehydration, lethargy, and anorexia and combined with respiratory exhaustion, which poses a serious threat to life. Generally, it needs to enter ICU for treatment [3^,^^4^].

Severe pneumonia is a common acute and critical disease, and it is also a common disease in ICU [5]. Its condition is serious, and its mortality is high. How to control the occurrence and development of severe pneumonia is one of the difficult problems that perplex the medical workers in the department of critical medicine [6^,^^7^]. To control severe pneumonia, we must first control pneumonia, find the risk factors of pneumonia, and prevent the development of pneumonia to severe pneumonia which is an important measure.

It is reported that the risk of death in patients with severe pneumonia is usually related to the following risk factors: aerobic Gram-negative bacterial infection, especially *Pseudomonas aeruginosa* infection, the severity of basic diseases, aging, inappropriate antimicrobial treatment, shock, malignant tumors, bilateral pulmonary infiltrative shadows, the application of a large number of antibiotics, long-term hospitalization, mechanical ventilation treatment, etc. [8^,^^9^]. During treatment, the course of the disease changes rapidly, and the course of the disease changes rapidly. Timely treatment and nursing are very important [10–12].

The article "Analysis of Risk Factors for Pneumonia Death in ICU Environment Based on Logistic Regression" was retracted in 2023. Reasons: signs of a paper mill; suspected computer-generated content; unreliable results or conclusions; lack of ethics approval or compliance.

The routine nursing mode provides nursing for the disease itself, but it pays insufficient attention to the emotional state of patients and other aspects, which leads to the loneliness and pessimism of ICU patients [13–16]. Therefore, nursing measures need to be improved. Systematic nursing provides emotional, dietary, ward environment, and other multiangle interventions to meet the physiological and psychological needs [17–20]. Therefore, high-quality nursing is very important in the treatment of patients with pneumonia.

Due to the limited research on the relationship between high-quality care and death caused by pneumonia, we will analyze the risk factors of death caused by pneumonia based on real-world data, especially the role of high-quality care in this process.

## 2. Methods

### 2.1. Patients' Information

In this research, we collected the basic information and nursing information of 80 patients with pneumonia in the department of critical medicine of the fourth hospital of Wuhan from January 2015 to January 2021. Among them, 40 patients died, and the other 40 patients survived and were discharged the basic information of patients includes: age, gender, marital status, education, residence, and nursing services obtained.

### 2.2. Evaluation of Quality Nursing

High-quality nursing is a nursing model that takes patients as the center, strengthens the basic nursing concept, deepens the connotation of nursing profession, comprehensively implements nursing responsibility, and improves the overall nursing service level. Compared with traditional nursing, it pays more attention to the needs of patients. In recent years, high-quality nursing has been widely used in general surgery, critical care department, and other departments. In critical care department, only the impact on patients' psychology and prognosis has been widely studied [21^,^^22^].

### 2.3. Statistical Analysis

In the baseline data analysis, Chi-square test and *t*-test were used to analyze the difference of demographic and social economic data in two groups, respectively.

Subsequently, we used Pearson's correlation matrix to identify related factors associated with pneumonia patients living status. After that, we conducted a logistic regression to find out significant risk factors for living status of pneumonia patients and calculating odds ratios (OR) values. All the analyses were conducted in the R software 4.1.2 (the R Foundation for Statistical Computing, USA). Two-sided *P* < 0.05 was considered statistically significant. All continuous variables were described as mean ± standard deviation.

The article "Analysis of Risk Factors for Pneumonia Death in ICU Environment Based on Logistic Regression" was retracted in 2023. Reasons: signs of a paper mill; suspected computer-generated content; unreliable results or conclusions; lack of ethics approval or compliance.

### 2.4. Logistic Regression

Logistic regression was a supervised learning algorithm used to predict a dependent categorical target variable. In essence, if you had a large set of data that you want to categorize, logistic regression might be able to help.

The principle of the logistic regression could be summarized as follows [23]:

Binary logistic regressions estimated the likelihood that a characteristic of a binary variable was present, given the values of the covariates. Suppose *Y* was a binary response variable where *Y*_*i*_ = 1 if the character was present and *Y*_*i*_ = 0 if the character was absent and the data [*Y*_1_, *Y*_2_, ⋯, *Yn*] were independent. Let *π*_*i*_ be the probability of success. Additionally, consider *x* = (x_1_, x_2_, ⋯, x_p_) as a set of explanatory variables which can be discrete, continuous, or a combination of both discrete and continuous. Then, the logistic function for *π*_*i*_ was given by

(1) $$\begin{array}{c} \log\text{it}\left(\pi_{i}\right)=\beta_{0}+\beta_{1}x_{i1}+\beta_{2}x_{i2}+\cdots +\beta_{p}x_{i}{,}_{p};. \end{array}$$

Here, *π*_*i*_ denoted the probability that a sample was in a given category of the dichotomous response variable, commonly called as the “success probability” and, clearly, 0 ≤ *π*_*i*_ ≤ 1. (*π*_*i*_/(1 − *π*_*i*_)) was called the odds ratio or relative risk.

## 3. Results

The results of pneumonia patients demographic data showed that the sample was comprised of the elderly in death group (89.7 ± 8.37 years old) and living group (84.1 ± 8.21 years old), male in death group (*n* = 25, 62.5%), male in living group (*n* = 29, 72.5%), predominantly married in living group (*n* = 27, 69.2%), widowed in death group (*n* = 21, 53.8%), no education in death group (*n* = 16, 40.0%) and living group (*n* = 11, 27.5%), rural area in both dead and live groups (*n* = 35, 87.5%) with general nursing in death group (*n* = 24, 60.0%), and high-quality nursing (*n* = 25, 65.5%) (Table 1). In the differences analysis of the baseline data, only age showed significant difference among two status groups, which demonstrated that two groups had good comparability.

After exploratory analysis, Pearson's correlation matrix analysis was conducted for the correlation of 7 variables for the further logistic regression (Figure 1). According to the matrix, there was correlation between living status, age, and marriage (the correlation value is -0.26 for age and 0.18 for marriage, *P* < 0.05). Exploratory factor analysis confirmed limited correlated covariant, which was a good basis for logistic regression.

The article "Analysis of Risk Factors for Pneumonia Death in ICU Environment Based on Logistic Regression" was retracted in 2023. Reasons: signs of a paper mill; suspected computer-generated content; unreliable results or conclusions; lack of ethics approval or compliance.

To further analyze the risk level of 6 factors, we conducted the logistic regression (Table 2). The living of pneumonia patients were related with age (*β* = −0.066, *P* = 0.047), no education (*β* = −1.58, *P* = 0.042), and high-quality nursing (*β* = 1.01, *P* = 0.034), respectively. Furthermore, model OR results showed that age (OR = 0.94) and no education (OR = 0.21) might be harmful for pneumonia patients living status while high-quality nursing (OR = 2.72) might be helpful for pneumonia patients living status.

## 4. Discussion

Based on our analysis results, we could see that high-quality care was an important factor to help ICU patients with pneumonia survival (OR = 2.72) and had a strong intervention effect. The high-quality nursing group used modular nursing intervention, as follows [2^,^^13^]: (1) oxygen supply nursing module: nurses paid close attention to the patient's oxygen supply status, controlled the oxygen supply concentration, and reduced the oxygen supply concentration when the patient was found to have carbon dioxide retention, so as to avoid fainting. (2) In respiratory tract care module, they pay close attention to the patient's sputum state. If the patient's sputum was thick and cannot be automatically discharged from the mouth, it was necessary to give mechanical ventilation to keep the patient's airway moist to avoid blockage, given the patient with cough difficulty body position drainage to assist in the discharge of sputum and perform sputum suction intervention when necessary. (3) In psychological counseling module, they strengthen communication with patients who were awake, encourage patients to state their feelings, doubts, and concerns, and used their professional knowledge to comfort patients to alleviate their bad emotions caused by diseases. In the process of communication, patients could be appropriately massaged to increase their comfort. For patients who have been in coma, regular limb massage was needed to enhance the soothing effect and stimulate their brain nerves. (4) In complication nursing module, during the treatment process, nurses should pay close attention to the changes of lip color and skin color of patients, especially older patients, who were generally complicated with basic diseases and were more likely to have related complications. When patients had cyanosis of lips and pale complexion, they should timely inform doctors for treatment to avoid complications such as heart failure and circulatory disorders.

The article "Analysis of Risk Factors for Pneumonia Death in ICU Environment Based on Logistic Regression" was retracted in 2023. Reasons: signs of a paper mill; suspected computer-generated content; unreliable results or conclusions; lack of ethics approval or compliance.

In addition to the effective help of high-quality care for patients with pneumonia, age had a strong correlation with the death of patients with pneumonia (OR = 0.94). It was reported that there were many risk factors for severe pneumonia. The incidence rate of elderly patients was high, which was related to the poor nutritional status of elderly people, more chronic diseases, neuromuscular diseases, and low immune function. Through research, it was found that age > 75 was one of the risk factors for nosocomial infection. This conclusion was consistent with our analysis [24–28].

In addition, uneducated patients also had a strong relationship with the death of patients with pneumonia (OR = 0.21). At present, there were few reports on this result. Maybe this was a direction worthy of further research. The education level of patients had a strong relationship with the outcome of death, suggesting the importance of basic education, which was also an important part of social intervention [29–32].

## 5. Conclusion

In conclusion, quality care played an important protective role in the survival of patients with pneumonia, and old age and uneducated might be the risk factors for the death of patients with pneumonia. However, there were several limitations in our research; firstly, the design of this study was based on case-control not cohort, which might be not enough for causal relationship. Secondly, the study samples were limited and study center is not multiple, which could be considered in the future.

## Figures and Tables

**Figure 1:** Correlation matrix of included variables.

**Table 1:** Demographic information of included individuals.

	Dead (*N* = 40)	Live (*N* = 40)	*P* value for *t* or Chi-square test
Age	89.7 ± 8.37	84.1 ± 8.21	0.004
Gender			0.474
Female	15 (37.5%)	11 (27.5%)	
Male	25 (62.5%)	29 (72.5%)	
Marriage status			0.018
Divorced	1 (2.57%)	1 (2.56%)	
Married	16 (41.0%)	27 (69.2%)	
Not applicable	2 (5.13%)	2 (5.13%)	
Widowed	21 (53.8%)	10 (25.6%)	
Education			0.247
Not graduated from primary school	6 (15.0%)	9 (22.5%)	
Collage or above	1 (2.50%)	2 (5.00%)	
High school	4 (10.0%)	2 (5.00%)	
Middle school	11 (27.5%)	8 (20.0%)	
No education	16 (40.0%)	11 (27.5%)	
Primary school	2 (5.00%)	8 (20.0%)	
Residence			1
Rural	35 (87.5%)	35 (87.5%)	
Urban	5 (12.5%)	5 (12.5%)	
Nursing			0.07
High-quality nursing	16 (40.0%)	25 (62.5%)	
General nursing	24 (60.0%)	15 (37.5%)	

**Table 2:** Logistic regression of risk factors for pneumonia patients death.

	*β*	Std. error	OR	*P* value
Age	-0.066	0.036	0.94	0.047^∗^
Male	0.84	0.66	2.31	0.21
Married	-14.19	1455.39	0.005	0.99
Marriage or widowed	-15.69	1455.39	0.006	0.99
Collage or above	2.09	1.91	8.07	0.27
High school	-0.44	1.2	0.64	0.71
Middle school	-0.53	0.87	0.59	0.54
Primary school	1.12	1.07	3.06	0.29
No education	-1.58	0.88	0.21	0.042^∗^
Urban	-0.63	0.98	0.54	0.45
High-quality nursing	1.01	0.58	2.72	0.034^∗^

^∗^ *P* < 0.05, model coefficient significance.

The article "Analysis of Risk Factors for Pneumonia Death in ICU Environment Based on Logistic Regression" was retracted in 2023. Reasons: signs of a paper mill; suspected computer-generated content; unreliable results or conclusions; lack of ethics approval or compliance.

## Data Availability

The datasets used and analyzed during the current study are available from the corresponding author upon reasonable request.
